The article "Preliminary Study on Risk Factors for Morbidity of Nonalcoholic Fatty Liver Disease in High-Income Male Population" was retracted in 2023. Reasons: signs of a paper mill; compromised peer review; unreliable results or conclusions.

# Preliminary Study on Risk Factors for Morbidity of Nonalcoholic Fatty Liver Disease in High-Income Male Population

**DOI:** 10.1155/2022/9331284

**Published:** 2022-02-23

**Authors:** Li Han, Yuting Zhang, Cui Yue, Yiqin Huang, Yumin Wu, Jie Chen

**Affiliations:** ^1^Huadong Hospital Affiliated to Fudan University, Department of Traditional Chinese Medicine, 221 Yan'an West Road,Jing'an District, Shanghai 200040, China; ^2^Huadong Hospital Affiliated to Fudan University, Department of Digestion, 221 Yan'an West Road,Jing'an District, Shanghai 200040, China; ^3^The Office of Good Clinical Practice, 221 West Yan'an Road, Huadong Hospital, Shanghai 200040, China; ^4^Huadong Hospital Affiliated to Fudan University, Department of Nephrology, 221 Yan'an West Road,Jing'an District, Shanghai 200040, China; ^5^Huadong Hospital Affiliated to Fudan University, Department of Geriatrics, 317 Room,168 Yan'an West Road,Jing'an District, Shanghai 200040, China

## Abstract

**Objectives:**

Believed to be a result of metabolic syndrome and unhealthy lifestyle, the incidence of nonalcoholic fatty liver disease (NAFLD) has become a serious public health problem. Among the high-income male population, metabolic syndrome and unhealthy lifestyle are particularly prominent. Therefore, we conducted a survey on 375 high-income male subjects, expecting to understand the risk factors and related factors for morbidity of NAFLD among the high-income male population being physically examined in Shanghai.

**Methods:**

A cross-sectional study was applied to 375 high-income male subjects (including 190 patients with NAFLD and 185 non-NAFLD subjects) who were examined in the special needs clinic at Huadong Hospital affiliated to Fudan University. In combination with medical history, physical examination, and laboratory test results and by use of a self-made NAFLD health questionnaire, the basic data of the research objects were collected and the obtained data were subject to a correlation analysis.

**Results:**

This study investigated 375 high-income males, and the morbidity rate of NAFLD was 50.67%. The NAFLD group was higher than the non-NAFLD group in terms of body weight, BMI, systolic blood pressure, and diastolic blood pressure (*P* < 0.05). Hypertension (OR = 2.944), diabetes (OR = 7.278), and hyperuricemia (OR = 1.922) are the risk factors for NAFLD; compared with no metabolic diseases, one (OR = 1.848), two (OR = 2.417), and three metabolic diseases (OR = 14.788) are risk factors for the development of NAFLD. Compared with the non-NAFLD group, the NAFLD group had a higher level of WBC, RBC, Hb, PLT, FPG, HbA1c, ALT, AST, GGT, ALP, TP, and UA (*P* < 0.05). There was a statistically significant difference in the intake of supper and staple foods between the NAFLD group and the non-NAFLD group, and the highly greasy diet was a risk factor for NAFLD (OR = 2.173) as opposed to the nongreasy diet.

The article "Preliminary Study on Risk Factors for Morbidity of Nonalcoholic Fatty Liver Disease in High-Income Male Population" was retracted in 2023. Reasons: signs of a paper mill; compromised peer review; unreliable results or conclusions.

**Conclusion:**

High-income male population is a high-risk group of NAFLD. Most of the patients with NAFLD have abnormal biochemical indicators as opposed to the healthy population and are more likely to be complicated with other chronic diseases or abnormal health status. And the occurrence of hypertension, diabetes, and hyperuricemia is the risk factor for the development of NAFLD. At the same time, the number of metabolic diseases complicated is also a risk factor for NAFLD as compared with the absence of complications with such metabolic diseases. Compared with a diet that is not greasy, the fact that high-income male NAFLD patients have a very greasy diet increases the risk of NAFLD.

## 1. Introduction

Nonalcoholic fatty liver disease (NAFLD) has become the most common chronic liver disease worldwide. This is a disease that is thought to be closely related to obesity, insulin resistance, and genetic factors, including nonalcoholic simple steatosis and nonalcoholic steatohepatitis (NASH), and it may also develop into cirrhosis and liver cancer [1]. At present, NAFLD has become a common chronic hepatic pathological change in the world, and it has also gradually become the main cause of the discovery of liver enzyme abnormalities in chronic liver diseases and physical examinations [2]. Presently speaking, the prevalence rate of NAFLD varies from region to region and from population to population, ranging from 6.3% to 45% [3], and the prevalence of NAFLD in men is significantly higher than that in women. The rising impact of perioperative sonography is dependent on high-quality ultrasound systems. Ultrasonography examination is noninvasive and painless imaging that helps promote the analysis of abdominal [4]. A fatty liver-related meta-analysis in 2015 [5] showed that the prevalence of NAFLD in Chinese men was 19.28%, which was significantly higher than that in Chinese women (14.1%).

The pathogenesis of NAFLD has currently not yet been fully elucidated. It is currently believed that NAFLD is how metabolic syndrome manifests in the liver, and NAFLD is closely related to risk factors that are associated with metabolic syndrome and IR, including high fat, high-carbohydrate diet, sedentary, and insufficiently active lifestyles. At present, the results of several studies have shown that, among the risk factors of occurrence of NAFLD, unhealthy lifestyle plays an important role, and improving the lifestyle of patients with NAFLD can improve the disease status of patients with NAFLD [6].

The article "Preliminary Study on Risk Factors for Morbidity of Nonalcoholic Fatty Liver Disease in High-Income Male Population" was retracted in 2023. Reasons: signs of a paper mill; compromised peer review; unreliable results or conclusions.

However, with the development of society and the improvement of people's living standards, their lifestyles are gradually changing. There are some studies [7] reporting that, in 2016, the percentage of people with insufficient physical activity in high-income countries was 36.8%, which is more than two times the percentage of people with insufficient activity in low-income countries, and the lack of activity has been aggravated all along. Another study [8] also reported that, in China, among the population with high income, the meat, eggs, and milk are excessively consumed, and the incidence of chronic diseases among it was higher than that among the lower-income population. However, there is a lack of study on the correlation between the prevalence of NAFLD in the high-income population and their lifestyle characteristics. Therefore, we conducted a survey on the high-income male population in the special physical examination department of our hospital in terms of general health basic condition, blood test, abdominal B-ultrasound, and so on and collected their lifestyles in order to understand the health condition, the characteristics of blood indicators, dietary structure, exercise, and other conditions of NAFLD patients so as to further understand how the change of lifestyle, especially the change of dietary structure, affects NAFLD.

## 2. Method

This study included high-income males coming from the enterprise and public institution who received health examination at the special needs clinic and special needs medical department of Huadong Hospital affiliated to Fudan University from January 1, 2017, to December 31, 2017. According to the statistics about the income level in Shanghai released by the China Bureau of Statistics in Shanghai in 2017 and China's fiscal policy report of 2018 [9], we defined the population with an annual income that is more than or equal to 400,000 yuan as a high-income group. In this study, patients with severe cardiac insufficiency, renal insufficiency, respiratory failure, chronic infectious diseases, and complication with the secondary factors that can cause appetite and weight changes, such as Cushing's syndrome, pituitary dysfunction, and thyroid dysfunction, or the population who had a recent use of drugs such as steroids were excluded from this study because the disease the patients had may disturb their lifestyles [10]; for the same reason, the individuals who have intentionally lost weight or gained weight in the past three months were also not included in the study. Taking into consideration the fact that certain diseases may affect patients' B-ultrasound and blood test results, the patients with malignant tumors, patients with liver diseases other than NAFLD such as autoimmune liver disease, drug-induced liver disease, and viral hepatitis, and the individuals who take an amount of ethanol more than 140 g/week were also excluded [11, 12]. In addition, because this study requires full communication with participants about their lifestyles, we also excluded individuals who are incapable of normal communication and exchange.

The article "Preliminary Study on Risk Factors for Morbidity of Nonalcoholic Fatty Liver Disease in High-Income Male Population" was retracted in 2023. Reasons: signs of a paper mill; compromised peer review; unreliable results or conclusions.

### 2.1. Research Methods

The subjects included in the study were investigated, mainly including the personal data, physical examination, biochemical tests, and abdominal B-ultrasound regarding the subjects.

#### 2.1.1. Personal Data

Personal data included name, gender, age, past history (including the history of hypertension, hyperglycemia, hyperlipidemia, and hyperuricemia), and personal history. The diagnostic criteria for related complications in past history were as follows.

#### 2.1.2. Physical Examination

The subjects' height, weight, and blood pressure (BP) were measured:

1. Height and weight: the height and weight measurements were done with a calibrated height and weight meter. The measurement requires that the subjects of medical examination be fasting in the morning, empty the bladder, remove the excess accessories, take off the shoes, and wear a single-layer dress for measurement. The height and weight were both measured twice and the mean was taken; the height was measured in centimeters and the weight was measured in kilograms. Body mass index (BMI = weight (kg)/height (*m*)^2^) was calculated based on height and weight [12].
2. Blood pressure: blood pressure was measured according to the method of measuring blood pressure in the clinic room stated in the *Guideline for Prevention and Treatment of Hypertension in China 2010* [13, 14]. The subject rests at least 5 minutes quietly, then takes the sitting position, and places the upper arm at the level of the heart. The validated electronic blood pressure meter is used to measure the blood pressure of the upper arm of the subject, taking the side with a higher blood pressure reading as the measurement side, it is measured again after 1–2 minutes, the average of the two readings was taken as the result, if the difference between the two readings is found greater than 5 mmHg, then measure it again after 1–2 minutes, and the average of three readings was taken as the result.

#### 2.1.3. Biochemical Test

The medical examinee stops eating and drinking water after 20:00 on the night before blood sampling, and the upper limb venous blood is sampled for detection in the morning. The test contents include white blood cells (WBC), red blood cells (RBC), hemoglobin (Hb), platelets (PLT), Glycated hemoglobin (HbA1c), alanine aminotransferase (ALT), aspartate aminotransferase (AST), glutamyl transferase (GGT), alkaline phosphatase (ALP), total bilirubin (TBil), creatinine (Cr), uric acid (UA), triglyceride (TG), total cholesterol (TC), high-density lipoprotein (HDL-C), and low-density lipoprotein (LDL-C). All indicators are tested by the Department of Clinical Laboratory of Huadong Hospital affiliated to Fudan University.

The article "Preliminary Study on Risk Factors for Morbidity of Nonalcoholic Fatty Liver Disease in High-Income Male Population" was retracted in 2023. Reasons: signs of a paper mill; compromised peer review; unreliable results or conclusions.

#### 2.1.4. Abdominal Ultrasound Examination

All subjects underwent abdominal B-ultrasound examination on a fasting condition. The examination was performed by the sonographer using the same ultrasound apparatus. The imaging diagnostic criteria were based on the *Guidelines for Management of Nonalcoholic Fatty Liver Disease: An Updated and Revised Edition* [11].

#### 2.1.5. Filling of the Health Questionnaire

The self-designed health questionnaire was used to collect the data of the subjects, including basic conditions, exercise status, smoking and drinking, dietary habit, exercise, and chronic diseases. The health questionnaire is detailed in Appendix A.

### 2.2. Diagnostic Criteria

The diagnostic criteria of this study were based on the *Guidelines for Management of Nonalcoholic Fatty Liver Disease: An Updated and Revised Edition* [11].

### 2.3. Statistical Analysis

Statistical analysis was performed on relevant parameters using SPSS22.0. Firstly, the relevant parameters were subject to a normality test. The continuous measurement data that were normally distributed were described with the mean ± standard deviation, and an independent sample *t*-test was used for analysis. The skewness data were expressed as *M* (P25; P75); the nonparametric rank-sum test was used for comparison between groups; the statistical data were counted and analyzed by *χ*^2^ test; the analysis on the correlation between risk factors and NAFLD was performed using unconditional logistic regression analysis; the variable assignment is shown in Appendix B; odds ratio (OR) and its 95% confidence interval (95%CI) were calculated; if *P* < 0.05, the difference was considered statistically significant.

## 3. Results

This study investigated 375 subjects. The average age was 48.90 ± 6.05 years (range 33–61 years), and NAFLD patients were 190 with a prevalence rate of 50.67% (Table 1).

Compared with the non-NAFLD group, the NAFLD group had higher body weight, BMI, systolic blood pressure, and diastolic blood pressure than the non-NAFLD group, and the difference was statistically significant. The levels of white blood cells (WBC), red blood cells (RBC), hemoglobin (Hb), platelet (PLT), fasting plasma glucose (FPG), glycosylated hemoglobin (HbA1c), alanine aminotransferase (ALT), aspartate aminotransferase (AST), glutamyl transferase (GGT), alkaline phosphatase (ALP), total protein (TP), and uric acid (UA) were higher in NAFLD group, and the difference was statistically significant (*P* < 0.05). Other indicators between the two groups were not significantly different (Table 2).

*χ* ^2^ test results showed that the prevalence of hypertension, diabetes mellitus, hyperuricemia, and the number of combined metabolic diseases in the NAFLD group were significantly different from those in the non-NAFLD group (Table 3).

*χ* ^*2*^ test results showed that there was no significant difference between the NAFLD group and the non-NAFLD group in daily exercise, dining out, overeating, pressure feeding, eating before bedtime, and not eating breakfast. There was no significant difference in the number of bad habits between the two groups (Table 4). The composition of the three meals of the previous day before physical examination in the two groups is shown in Table 5. There was a significant difference in dinner intake between the NAFLD group and the non-NAFLD group (*P*=0.003). Meantime, the intake of staple food such as rice noodles in the NAFLD group was 300 g (237.50 g–400.00 g) one day before physical examination, and that of staple food intake in the non-NAFLD group was 300 g (200.00 g–300.00 g) one day before physical examination. The difference was statistically significant (*P* < 0.001).

The article "Preliminary Study on Risk Factors for Morbidity of Nonalcoholic Fatty Liver Disease in High-Income Male Population" was retracted in 2023. Reasons: signs of a paper mill; compromised peer review; unreliable results or conclusions.

Single-factor logistic regression analysis showed that BMI = 24–28 kg/m^2^ (*OR* = 2.657; 95%CI (1.654–4.267)) and BMI > 28 kg/m^2^ (*OR* = 13.333; 95%CI (5.984–29.709)) all increased the risk of NAFLD compared with BMI < 24 kg/m^2^. Hypertension (*OR* = 2.944; 95%CI (1.721–5.034)), diabetes (*OR* = 7.278; 95%CI (1.631–32.488)), and hyperuricemia (*OR* = 1.922; 95%CI (1.245–2.966)) were all risk factors for NAFLD. Compared with nonmetabolic diseases, one combined metabolic disease (*OR* = 1.848; 95%CI (1.096–3.117)), two combined metabolic diseases (*OR* = 2.417; 95%CI (1.334–4.380)), and three combined metabolic diseases (*OR* = 14.788; 95%CI (4.141–52.803)) increased the risk of NAFLD. The very greasy diet increased the risk of NAFLD compared with the nongreasy diet (*OR* = 2.173; 95%CI (1.187–3.978)) (Table 6).

BMI, hypertension, diabetes mellitus, hyperuricemia, the number of complications, and the intake of greasy diet were selected as candidate covariates by single-factor logistic regression, and the occurrence of NAFLD was taken as a dependent variable. The results of multivariate logistic stepwise regression analysis were as shown in Table 7. Compared with BMI < 24 kg/m^2^, BMI = 24–28 kg/m^2^ (*OR* = 2.406; 95%CI (1.453–3.986)), and BMI > 28 kg/m^2^ (*OR* = 12.463; 95%CI (5.412–28.699)) all increased the risk of NAFLD; compared with the nongreasy diet, the very greasy diet was a risk factor for NAFLD (*OR* = 2.184; 95%CI (1.102–4.327)).

The article "Preliminary Study on Risk Factors for Morbidity of Nonalcoholic Fatty Liver Disease in High-Income Male Population" was retracted in 2023. Reasons: signs of a paper mill; compromised peer review; unreliable results or conclusions.

According to the results of epidemiological investigation, the incidence of NAFLD is related to age. Variable age was included in the model, and multivariate logistic stepwise regression was used to consider metabolic complications, including hypertension, diabetes mellitus, and hyperuricemia, so no specific diseases were included. As shown in Table 8, compared with BMI＜24 kg/m^2^, BMI = 24–28 kg/m^2^ (*OR* = 2.552; 95%CI (1.540–4.231)) and BMI＞28 kg/m^2^ (*OR* = 13.642; 95%CI (5.856–31.780)) increased the risk of NAFLD incidence. Compared with the nongreasy diet, the very greasy diet increased the risk of NAFLD incidence (*OR* = 2.325; 95%CI (1.171–4.615)).

## 4. Discussion

The pathological features of NAFLD are steatosis of hepatocytes in the liver, with balloon-like changes of hepatocytes, mixed inflammatory cell infiltration in lobules, and perisinusoidal fibrosis [15]. The primary manifestation of the disease is nonalcoholic simple steatosis of the liver in the early stage, which can gradually develop into nonalcoholic steatohepatitis (NASH) and even cirrhosis and liver cancer. The prevalence of NAFLD varies from 6.3% to 45% in different regions and populations, with the prevalence of NASH ranging from 10% to 30% [3]. At present, the pathogenesis of NAFLD is not fully understood, but the working hypothesis of “double-hit” put forward in 1998 is widely accepted [16]. At present, the pathogenesis of NAFLD has been constantly improved, and the “ double-hit ” has gradually changed to the “multiple-hits” theory. However, insulin resistance still plays an important role in the pathogenesis of NAFLD. Generally speaking, the development stage and severity of NAFLD can be assessed by NAS score and staging of liver fibrosis, and the degree of hepatic steatosis can also be classified into three grades: mild, moderate, and severe by noninvasive B-mode ultrasonography and other imaging methods [16, 17]. However, the number of cases included in this study is relatively fewer, the discussion of grading may lead to large deviations, and this study is only a preliminary study, so we do not discuss further the relationship between the degree of liver fat infiltration and risk factors.

With the improvement of people's income level, the incidence of fatty liver is also rising year by year. NAFLD diagnosed by ultrasound has increased from 15% to 31% in the past 10 years [18]. A systematic review of global NAFLD morbidity assessment shows that the higher the economic status of countries, the higher the prevalence of NAFLD and the incidence of NAFLD in economically developed coastal areas is also higher than that in inland areas [19]. However, there is no unified annual income standard for the determination of high-income people in China. At present, some studies define the high-income group as the people whose annual income is more than 120,000 yuan, but this standard is obviously not suitable for Shanghai residents [20, 21]. According to China's fiscal policy report in 2018, the per capita disposable income of the middle-income group was 22495 yuan in 2017, while that of the high-income group was 64934 yuan [9]. It suggests that high-income males are high-risk groups of NAFLD, and we should pay great attention to the treatment and prevention of NAFLD in this part of the population. Considering the reasons, on the one hand, high-income people are basically mental workers, usually with less exercise, more bad diet, and living habits, which are risk factors for NAFLD. On the other hand, the prevalence of NAFLD in males is usually higher than that in females. Li reported that the prevalence of NAFLD was 24.81% in males and 13.16% in females [22]. The possible reasons are as follows. Males have a larger proportion of unhealthy lifestyles than females, such as overeating, smoking, and drinking, more risk factors for NAFLD, so the incidence of NAFLD is higher [13]. Second, the protective effect of estrogen on NAFLD: estrogen can regulate blood lipid metabolism and intrahepatic fat distribution; it can ameliorate NAFLD [23]. Relevant literature also proves that the prevalence of NAFLD in premenopausal women is lower than that in men, while the prevalence of postmenopausal women can be significantly increased, even higher than that in men [5]. This may be related to the decrease of estrogen level and the relative increase of androgen level in postmenopausal women. Third, the effect of androgen on adiponectin secretion: adiponectin is a protein secreted by adipocytes, which can inhibit inflammation of the liver and delay fibrosis of liver tissue [24]. Nishizawa also found that androgen can reduce plasma adiponectin levels [25]. Androgen level in males is higher than that in females, and plasma adiponectin level is lower, so the incidence of NAFLD is higher than that of women.

The article "Preliminary Study on Risk Factors for Morbidity of Nonalcoholic Fatty Liver Disease in High-Income Male Population" was retracted in 2023. Reasons: signs of a paper mill; compromised peer review; unreliable results or conclusions.

As a common liver disease, NAFLD often occurs not alone but always with obesity, hypertension, hyperlipidemia, hyperglycemia, and other metabolic diseases [2, 26]. Lonardo A even found that NAFLD could occur before metabolic syndrome and diabetes, further promoting the development of various metabolic diseases [18]. In this study, we found that the body weight, BMI, systolic, and diastolic blood pressure of the NAFLD group were higher than those of the non-NAFLD group, and the levels of fasting blood sugar, glycosylated hemoglobin, and uric acid of the NAFLD group were higher than those of the non-NAFLD group. After analysis, the results showed that BMI, hypertension, diabetes, hyperuricemia, and the number of metabolic diseases were risk factors for NAFLD, which was basically consistent with the known risk factors of NAFLD [3, 27]. The increase of ALT and GGT was positively correlated with metabolic syndrome and type 2 diabetes [5]. The 2018 edition of China's NAFLD treatment guidelines also showed that the increase of ALT, AST, and other indicators is a high-risk factor for NAFLD to further develop to NASH [28]. In this study, compared with the non-NAFLD group, the NAFLD group had higher levels of ALT, AST, GGT, and ALP, with statistical significance.

NAFLD and metabolic diseases have complex relationships with people's dietary structure, sports, and other lifestyles. Generally speaking, NAFLD patients exercise significantly less than healthy people. Lack of physical exercise, high fat intake, overeating, eating before bedtime, frequently eating out, and other bad diets and exercise habits are all risk factors for NAFLD [29, 30]. In this study, we found that no matter whether NAFLD occurs or not, high-income men have less exercise and more bad diet habits. No statistical correlation was found between daily exercise, catering service, overeating, pressure feeding, eating before bedtime, dining out, not eating breakfast, and the number of bad habits and the occurrence of NAFLD among high-income men. However, the reason may be that the sample selected in this study comes from the special need clinic physical examination population, mainly mental workers, less daily exercise, and greater work pressure. To some extent, it is similar to its working environment and daily living habits. On the other hand, evidence from many countries and areas shows that NAFLD patients have higher energy intake and generally higher fat and carbohydrate intake than healthy people [31–33]. In this study, we analyzed the three meals and total energy intake, staple food intake, and fat intake of the NAFLD group and the non-NAFLD group. The results showed that, among high-income men, compared with those non-NAFLD, NAFLD patients had a higher intake of dinner, and more people had high fat and carbohydrate intake. Logistic regression analysis also showed that, compared with the nongreasy diet, the greasy diet is a risk factor for NAFLD, which means that low carbohydrate and low-fat diets may improve the disease of NAFLD patients. At present, it is generally believed that the recommended diet for NAFLD patients should be based on the principle of low fat and carbohydrate and increasing dietary fiber intake [7, 34]. At present, China's national income is gradually increasing, and people's lifestyle and dietary structure are also undergoing major changes. The traditional diet is mainly high carbohydrate, but with the gradual increase of people's income, there is a gradual increase in oil intake [33], which requires us to recommend appropriate life intervention methods to these NAFLD patients according to their specific conditions in order to obtain better intervention results.

The article "Preliminary Study on Risk Factors for Morbidity of Nonalcoholic Fatty Liver Disease in High-Income Male Population" was retracted in 2023. Reasons: signs of a paper mill; compromised peer review; unreliable results or conclusions.

## 5. Conclusion

High-income male population is a high-risk group of NAFLD. Most of the patients with NAFLD have abnormal biochemical indicators as opposed to the healthy population and are more likely to be complicated with other chronic diseases or abnormal health status. In the future, it is emergence to diagnose the NAFLD early and come up with high-efficiency treatment options to improve patients' life.

## Figures and Tables

**Table 1:** Demographic compositions of NAFLD.

Age	Number	Morbidity rate (%)
30–39 y	15	33.3
40–49 y	199	52.26
50–59 y	145	51.03
60–69 y	16	43.75
Sum total	375	50.67

**Table 2:** Comparison of general conditions and biochemistry tests between the NAFLD group and the non-NAFLD group.

	NAFLD group (*n* = 190)	Non-NAFLD group (*n* = 185)	*P* value
Age (years)	49.24 ± 5.81	48.55 ± 6.28	0.273
Height (cm)	174.11 ± 5.21	173.89 ± 5.39	0.689
Weight (cm)	79.84 ± 11.15	72.00 ± 8.79	<0.001
BMI (kg/m^2^)	26.42 ± 2.76	23.80 ± 2.37	<0.001
Systolic blood pressure/SBP (mmHg)	121.73 ± 12.84	118.52 ± 13.76	0.020
Diastolic blood pressure/DBP (mmHg)	80.15 ± 9.12	78.13 ± 9.68	0.038
White blood cells/WBC (10^9^/L)	6.86 ± 1.59	6.47 ± 1.57	0.019
Red blood cells/RBC (10^12^/L)	5.05 ± 0.38	4.95 ± 0.37	0.009
Hemoglobin/Hb (g/L)	155.14 ± 9.83	152.48 ± 9.46	0.008
Platelet/PLT (10^9^/L)	239.94 ± 52.77	224.62 ± 46.50	0.003
Fasting plasma glucose/FPG (mmol/L)	5.20 (4.90,5.80)	5.00 (4.70,5.30)	0.000
Glycosylated hemoglobin/HbA1c (%)	5.50 (5.30,5.80)	5.40 (5.20,5.60)	0.003
Alanine aminotransferase/ALT (U/L)	27.00 (20.00,40.00)	20.00 (15.00,26.00)	0.000
Aspartate aminotransferase/AST (U/L)	21.00 (18.00,25.00)	20.00 (18.00,22.00)	0.002
Glutamyl transferase/GGT (U/L)	35.90 (24.87,54.55)	25.60 (18.95,37.30)	0.000
Alkaline phosphatase/ALP (U/L)	68.00 (58.00,77.25)	63.00 (54.00,75.50)	0.027
Total bilirubin/TBIL (*μ*mol/L)	12.10 (10.10,15.52)	11.80 (8.95,16.05)	0.687
Direct bilirubin/DBIL (*μ*mol/L)	4.60 (3.80,5.60)	4.80 (3.60,5.90)	0.961
Indirect bilirubin/IBIL (*μ*mol/L)	7.40 (5.77,9.90)	7.10 (5.20,10.50)	0.557
Total protein/TP (g/L)	75.33 ± 3.62	74.52 ± 3.66	0.032
Albumin/ALB (g/L)	49.22 ± 2.16	48.92 ± 2.32	0.208
Globulin/GLOB (g/L)	26.12 ± 3.21	25.60 ± 3.33	0.127
Albumin/globulin/A/G	1.91 ± 0.26	1.95 ± 0.29	0.262
Creatinine/Cr (*μ*mol/L)	85.00 (76.80,93.20)	86.60 (80.85,93.95)	0.129
Uric acid/UA (*μ*mol/L)	408.93 ± 80.50	372.37 ± 77.12	<0.001
Triglyceride/TG (mmol/L)	1.60 (1.20,2.30)	1.60 (1.10,2.10)	0.106
Total cholesterol/TC (mmol/L)	5.17 (4.61,5.72)	5.05 (4.42,5.63)	0.119
High-density lipoprotein-cholesterol/HDL-C (mmol/L)	1.36 ± 0.34	1.40 ± 0.30	0.260
Low-density lipoprotein-cholesterol/LDL-C (mmol/L)	3.04 ± 0.75	2.94 ± 0.84	0.223
Apolipoprotein A1/ApoA1 (g/L)	1.35 ± 0.23	1.38 ± 0.20	0.201
Apolipoprotein B/ApoB (g/L)	0.97 ± 0.20	0.93 ± 0.22	0.079
Alpha fetoprotein/AFP (g/L)	3.40 ± 1.70	3.37 ± 1.90	0.878

The article "Preliminary Study on Risk Factors for Morbidity of Nonalcoholic Fatty Liver Disease in High-Income Male Population" was retracted in 2023. Reasons: signs of a paper mill; compromised peer review; unreliable results or conclusions.

**Table 3:** Comparisons of related complications between the NAFLD group and the non-NAFLD group.

		NAFLD group (*n* = 190)	Non-NAFLD group (*n* = 185)	*χ* ^2^ value	*P* value
Hypertension (*n* = 79)		56 (29.47%)	23 (12.43%)	16.370	<0.001
Diabetes (*n* = 16)		14 (7.37%)	2 (1.08%)	7.597	0.006
Hyperlipidemia (*n* = 202)		108 (56.84%)	94 (50.81%)	1.372	0.241
Hyperuricemia (*n* = 129)		79 (41.58%)	50 (27.03%)	8.796	0.003
Number of combined metabolic diseases	0	33 (17.37%)	61 (32.97%)	26.212	<0.001
	1	82 (43.16%)	82 (44.32%)		
	2	51 (26.84%)	39 (21.08%)		
	≥3	24 (12.63%)	3 (1.62%)		

**Table 4:** Comparison of lifestyle between the NAFLD group and the non-NAFLD group.

			NAFLD group (*n* = 190)	Non-NAFLD group (*n* = 185)	*χ* ^2^ value	*P* value
Daily exercise	Basic inactivity		124 (65.26%)	130 (70.27%)	1.987	0.575
	Light volume exercise		46 (24.21%)	34 (18.38%)		
	Medium volume exercise		16 (8.42%)	16 (8.65%)		
	Mass volume exercise		4 (2.11%)	5 (2.70%)		
Bad eating habits	Overeating		79 (41.58%)	79 (42.70%)	0.049	0.826
	Pressure feeding		49 (25.79%)	34 (18.38%)	2.987	0.084
	Eating before bedtime		75 (39.47%)	85 (45.95%)	1.605	0.205
	Frequently dining out		56 (29.47%)	55 (29.73%)	0.003	0.957
	Not eating breakfast		17 (8.95%)	17 (9.19%)	0.007	0.935
	Number of bad eating habits	0	35 (18.42%)	26 (14.05%)	2.652	0.448
		1	79 (41.58%)	75 (40.54%)		
		2	49 (25.79%)	60 (32.43%)		
		≥3	27 (14.21%)	24 (12.97%)		

**Table 5:** Comparison of three meals composition between the NAFLD group and the non-NAFLD group.

	NAFLD group (*n* = 190)	Non-NAFLD group (*n* = 185)	*P* value
Breakfast (kcal)	500.00 (400.00,700.00)	500.00 (400.00,700.00)	0.674
Lunch (kcal)	600.00 (400.00,800.00)	700.00 (400.00,800.00)	0.223
Dinner (kcal)	700.00 (500.00,900.00)	700.00 (500.00,800.00)	0.003
Snack (kcal)	75.00 (0.00,162.50)	50.00 (0.00,20.00)	0.173
Total intake (kcal)	2000.00 (1675.00,2256.00)	1900.00 (1600.00,2200.00)	0.051

The article "Preliminary Study on Risk Factors for Morbidity of Nonalcoholic Fatty Liver Disease in High-Income Male Population" was retracted in 2023. Reasons: signs of a paper mill; compromised peer review; unreliable results or conclusions.

**Table 6:** Single-factor logistic regression for risk factors associated with NAFLD.

		*β*	*SE*	Wald *χ*^2^	*P* value	*OR* (95%CI)
Age groups	30–39 years					
	40–49 years	0.784	0.566	1.918	0.166	2.189 (0.722–6.637)
	50–59 years	0.725	0.572	1.647	0.199	2.085 (0.679–6.400)
	60–69 years	0.442	0.744	0.352	0.553	1.556 (0.362–6.690)
BMI	<24 kg/m^2^					
	24–28 kg/m^2^	0.977	0.242	16.323	<0.001	2.657 (1.654–4.267)
	>28 kg/m^2^	2.590	0.409	40.154	<0.001	13.333 (5.984–29.709)
Hypertension		1.080	0.274	15.547	<0.001	2.944 (1.721–5.034)
Hyperlipidemia		−0.243	0.208	1.370	0.242	0.784 (0.522–1.178)
Diabetes		1.985	0.763	6.763	0.009	7.278 (1.631–32.488)
Hyperuricemia		0.653	0.222	8.693	0.003	1.922 (1.245–2.966)
Number of combined metabolic diseases	0					
	1	0.614	0.267	5.310	0.021	1.848 (1.096–3.117)
	2	0.883	0.303	8.473	0.004	2.417 (1.334–4.380)
	≥3	2.694	0.649	17.208	<0.001	14.788 (4.141–52.803)
Daily exercise	Basic inactivity					
	Light volume exercise	0.350	0.259	1.826	0.177	1.418 (0.854–2.355)
	Medium to mass volume exercise	−0.002	0.337	0.000	0.996	0.998 (0.516–1.932)
Catering service in peacetime	Little					
	Commonly	−0.411	0.315	1.700	0.192	0.663 (0.357–1.230)
	Quite a lot	−0.198	0.294	0.453	0.501	0.821 (0.462–1.459)
Overeating		−0.046	0.209	0.049	0.826	0.955 (0.634–1.439)
Pressure feeding		0.434	0.252	2.954	0.085	1.543 (0.942–2.529)
Eating before bedtime		−0.265	0.209	1.603	0.206	0.767 (0.5.9–1.156)
Frequently dining out		−0.012	0.226	0.003	0.957	0.988 (0.634–1.539)
Not eating breakfast		−0.029	0.360	0.007	0.935	0.971 (0.480–1.965)
Number of bad habits	0					
	1	−0.208	0.310	0.447	0.504	0.812 (0.442–1.493)
	2	−0.351	0.325	1.165	0.280	0.704 (0.372–1.331)
	≥3	0.048	0.379	0.016	0.899	1.049 (0.499–2.206)
Intake stratification of carbohydrate	Little					
	Medium	0.552	0.431	1.637	0.201	1.737 (0.746–4.045)
	Mass	0.566	0.404	1.967	0.161	1.761 (0.799–3.884)
Dietary greasiness	Not greasy					
	Medium greasy	0.271	0.287	0.890	0.345	1.311 (0.747–2.300)
	Very greasy	0.776	0.309	6.321	0.012	2.173 (1.187–3.978)
Intake stratification of total energy	0–1400 kcal					
	1400–1800 kcal	−0.032	0.389	0.007	0.935	0.969 (0.452–2.075)
	1800–2200 kcal	0.347	0.370	0.880	0.348	1.415 (0.685–2.919)
	2200–2400 kcal	0.246	0.420	0.344	0.558	1.279 (0.561–2.916)
	>2400 kcal	0.572	0.425	1.817	0.178	1.772 (0.771–4.073)

**Table 7:** Multivariate logistic regression analysis of risk factors associated with NAFLD.

		*β*	*SE*	Wald **χ**^2^	*P* value	*OR* (95%CI)
BMI	<24 kg/m^2^					
	24–28 kg/m^2^	0.878	0.258	11.627	0.001	2.406 (1.453–3.986)
	＞28 kg/m^2^	2.523	0.426	35.138	＜0.001	12.463 (5.412–28.699)
Hypertension		0.664	0.390	2.895	0.089	1.943 (0.904–4.177)
Diabetes		1.386	0.860	2.596	0.107	3.999 (0.741–21.581)
Hyperuricemia		0.347	0.355	0.953	0.329	1.415 (0.705–2.839)
Number of combined metabolic diseases	0					
	1	0.506	0.313	2.621	0.105	1.659 (0.899–3.062)
	2	0.127	0.502	0.064	0.801	1.135 (0.424–3.039)
	≥3	1.435	0.926	2.398	0.121	4.198 (0.683–25.795)
Dietary greasiness	Not greasy					
	Medium greasy	0.221	0.325	0.462	0.497	1.248 (0.659–2.361)
	Very greasy	0.781	0.349	5.013	0.025	2.184 (1.102–4.327)

The article "Preliminary Study on Risk Factors for Morbidity of Nonalcoholic Fatty Liver Disease in High-Income Male Population" was retracted in 2023. Reasons: signs of a paper mill; compromised peer review; unreliable results or conclusions.

**Table 8:** Multivariate logistic regression analysis of risk factors associated with NAFLD.

		*β*	*SE*	Wald *χ*^2^	*P* value	*OR* (95%CI)
Age	30–39 years old					
	40–49 years old	1.134	0.620	3.348	0.067	3.108 (0.922–10.468)
	50–59 years old	1.080	0.626	2.980	0.084	2.946 (0.864–10.045)
	60–69 years old	0.921	0.840	1.201	0.273	2.511 (0.484–13.029)
BMI	<24 kg/m^2^					
	24–28 kg/m^2^	0.937	0.258	13.210	<0.001	2.552 (1.540–4.231)
	>28 kg/m^2^	2.613	0.431	36.375	<0.001	13.642 (5.856–31.780)
Number of combined metabolic diseases	0					
	1	0.689	0.297	5.403	0.020	1.992 (1.114–3.562)
	2	0.735	0.337	4.739	0.029	2.085 (1.076–4.040)
	≥3	2.561	0.683	14.065	<0.001	12.949 (3.396–49.378)
Dietary greasiness	Not greasy					
	Medium greasy	0.320	0.325	0.970	0.325	1.377 (0.728–2.604)
	Very greasy	0.844	0.350	5.813	0.016	2.325 (1.171–4.615)

**Table 9:** Relevant factor assignment table.

Variable	Name	Assignment
Group	Group	0 = non-NAFLD group; 1 = NAFLD group
Age group	Age group	1 = 30–39 years, 2 = 40–49 years, 3 = 50–59 years, 4 = 60–69 years
BMI	*X*_1_	1≤24 kg/m^2^, 2 = 24–28 kg/m^2^, 3≥28 kg/m^2^
Breath test	*X*_2_	0 = negative, 1 = positive
Hypertension	*X*_3_	0 = No, 1 = Yes
Hyperlipidemia	*X*_4_	0 = No, 1 = Yes
Diabetes	*X*_5_	0 = No, 1 = Yes
Hyperuricemia	*X*_6_	0 = No, 1 = Yes
Number of combined metabolic diseases	*X*_7_	0 = no combined metabolic diseases
		1 = 1 combined metabolic disease
		2 = 2 combined metabolic diseases
		3 = 3 or more combined metabolic diseases
Daily exercise	*X*_8_	1 = basic inactivity, 2 = a little exercise, 3 = medium volume exercise, 4 = mass exercise
Catering service in peacetime	*X*_9_	1 = seldom, 2 = sometimes, 3 = often
Overeating	*X*_10_	0 = No, 1 = Yes
Eating when stressed	*X*_11_	0 = No, 1 = Yes
Eating before sleeping	*X*_12_	0 = No, 1 = Yes
Eating out often	*X*_13_	0 = No, 1 = Yes
No breakfast	*X*_14_	0 = No, 1 = Yes
Number of bad eating habits	*X*_15_	0 = No bad dietary habits
		1 = 1 bad dietary habits
		2 = 2 bad dietary habits
		3 = 3 or more bad dietary habits
Carbohydrate intake (calculated as the ratio of carbohydrate energy to daily energy intake)	*X*_16_	1≤26%, 2 = 26%–45%, 3≥45%
Dietary greasiness	*X*_17_	1 = not greasy, 2 = medium greasy, 3 = very greasy
Total energy intake stratification	*X*_18_	1 = 0–1400 kcal/d, 2 = 1400–1800 kcal/d, 3 = 1800–2200 kcal/d, 4 = 2200–2400 kcal/d, 5 ≥ 2400 kcal/d

The article "Preliminary Study on Risk Factors for Morbidity of Nonalcoholic Fatty Liver Disease in High-Income Male Population" was retracted in 2023. Reasons: signs of a paper mill; compromised peer review; unreliable results or conclusions.

## Data Availability

The data used to support this study are available from the corresponding author upon request.

## Appendix

### A. Health Questionnaire

Hello! Thank you very much for your participation in this survey. The purpose of this questionnaire is to understand your lifestyle and basic situation, so that medical staff can evaluate your situation and give suggestions. The information on the table only reflects your real situation, no right or wrong, and the information filled in the questionnaire will be absolutely confidential. The data will only be used for academic research. We will not transmit any personal information. Thank you for your participation (Table 9).

(i) Basic information
  (1) Name:
  (2) Age:
  (3) Gender: (①Men ②Women)
  (4) Height: cm, Weight: kg, Body mass index: kg/m^2^
  (5) Drink: (Yes, No, Occasionally) (beer, yellow wine, red wine, liquor) Amount Liang/Day, Total year. Smoke: (Yes, No) Cigarettes/Day, Total year.
  (6) Your personal income status:
  (<18000 Yuan/year, 18000–50000 Yuan/year, 50000–120000 Yuan/year, 120000–400000 Yuan/year, 400000–600000 Yuan/year, >600000 Yuan/year)
  Family composition:
  (7) Do you have any of the following diseases?
  ①Hypertension
  ②Diabetes
  ③Hyperlipidemia
  ④Hyperuricemia
  ⑤Other
  (ii) Please choose the following options according to your situation in the past month:
  (1) Do you often exercise? (Continuous exercise for more than half an hour a day)
  1 Basic inactivity (Exercise less than 1 day a week)
  2 A little exercise (Exercise 2-3 days a week)
  3 Medium volume exercise (Exercise 4-5 days a week)
  4 Mass exercise (Exercise more than 6 day a week)
  (2) Dietary habits:
      (1) What is your main diet? ①Meat dishes ②Vegetarian dishes ③Basic balance of meat and vegetable
      (2) Enjoy sweets (Yes, No)
      (3) The dishes are greasy? ①Little oil ②Commonly ③Greasy.
      (4) Do you overeat? ①Yes ②No
      (5) Do you have the habit of eating to relieve stress? ①Yes ②No
      (6) Do you often eat before sleeping? ①Yes ②No
      (7) Do you often eat out? ①Yes ②No
      (8) Do you often skip breakfast? ①Yes ②No
      (9) What kind of staple food do you usually eat? ①Rice ②Noodles ③Steamed buns ④Thin gruel, porridge ⑤Pancake ⑥Tubers ⑦Cake Daily staple food intake is about liang
      (10) Dining out for business or work: ① Seldom② Sometimes ③ Often
  (3) Eating on the latest day:
      Breakfast gram; gram; gram; Dining type
      Chinese food: staple food() gram; meat dishes() gram; gram vegetarian dishes
      (); gram; Dining type Dinner: staple food() gram; meat dishes
      () gram; gram vegetarian dishes(); gram; Dining type
      Other food intake kcal
  (1) Do you often exercise? (Continuous exercise for more than half an hour a day)
      1 Basic inactivity (Exercise less than 1 day a week)
      2 A little exercise (Exercise 2-3 days a week)
      3 Medium volume exercise (Exercise 4-5 days a week)
      4 Mass exercise (Exercise more than 6 day a week)
  (2) Dietary habits:
      (1) What is your main diet? ①Meat dishes ②Vegetarian dishes ③Basic balance of meat and vegetable
      (2) Enjoy sweets (Yes, No)
      (3) The dishes are greasy? ①Little oil ②Commonly ③Greasy.
      (4) Do you overeat? ①Yes ②No
      (5) Do you have the habit of eating to relieve stress? ①Yes ②No
      (6) Do you often eat before sleeping? ①Yes ②No
      (7) Do you often eat out? ①Yes ②No
      (8) Do you often skip breakfast? ①Yes ②No
      (9) What kind of staple food do you usually eat? ①Rice ②Noodles ③Steamed buns ④Thin gruel, porridge ⑤Pancake ⑥Tubers ⑦Cake Daily staple food intake is about liang
      (10) Dining out for business or work: ① Seldom② Sometimes ③ Often
  (3) Eating on the latest day:
      Breakfast gram; gram; gram; Dining type
      Chinese food: staple food() gram; meat dishes() gram; gram vegetarian dishes
      (); gram; Dining type Dinner: staple food() gram; meat dishes
      () gram; gram vegetarian dishes(); gram; Dining type
      Other food intake kcal
